The article "Predictive Role of ADA in Bronchoalveolar Lavage Fluid in Making the Diagnosis of Pulmonary Tuberculosis" was retracted in 2014. Reasons: plagiarism; overlap with other authors' work.

# Predictive Role of ADA in Bronchoalveolar Lavage Fluid in Making the Diagnosis of Pulmonary Tuberculosis

**DOI:** 10.1155/2013/851518

**Published:** 2013-12-24

**Authors:** Fariba Binesh, Abolhassan Halvani

**Affiliations:** ^1^Department of Pathology, Shahid Sadoughi University of Medical Sciences, Yazd 8919337692, Iran; ^2^Mortaz Hospital, Kashani Street, Yazd 8915173143, Iran

## Abstract

Current diagnostic tests for tuberculosis (TB) are time-consuming. The aim of this study was to evaluate the diagnostic usefulness of ADA in bronchoalveolar lavage fluid in patients with pulmonary TB. A cross-sectional study was performed in Yazd, Iran, between 2009 and 2010. Patients suspected of pulmonary TB with negative sputum smear for AFB were included in the study. Mean ADA levels in BAL fluids were measured and compared between study groups. Sixty-three patients were enrolled in the study among which 15 cases had pulmonary TB, 33 had pulmonary diseases other than TB, and 15 subjects with normal bronchoscopy results were considered as controls. Mean ADA levels in BAL fluid were 4.13 ± 2.55, 2.42 ± 1.06, and 1.93 ± 0.88, respectively. This rate was significantly higher in the pulmonary TB group compared to the other two groups (*P* = 0.001). Using ROC curve with a cut-off value of 3.5 IU/L, the highest sensitivity (57%) and specificity (84%) were obtained in diagnosis of TB. The results showed that although ADA activity in BAL fluid of pulmonary TB patients was higher than those seen in other diseases, a negative test does not rule out pulmonary TB.

## 1. Introduction

Tuberculosis (TB) is the second most important cause of death from infectious diseases in the world [1]. It is a major public health problem in developing countries including Iran. Multidrug resistance in tuberculosis and its association with acquired immunodeficiency syndrome (AIDS) have further highlighted the importance of this disease. The diagnosis is usually based on clinical presentation, radiologic findings, and positive tuberculin and/or skin tests. However, clinicoradiological features are variable and the latter tests may be falsely negative. The gold standard of TB diagnosis requires the growth of Mycobacterium in specimen cultures, but the cultures are time-consuming and have low positivity rates, with a mean sensitivity of 43%–83% depending on the quality of samples cultured and methods utilized [2]. Since delay is unacceptable in emergency situations, it is necessary to find faster methods with higher sensitivity. The polymerase chain reaction (PCR) assay has shown good sensitivity and specificity in some studies [3], but it is not cost-effective and few centers use it in Iran. Several biomarkers like adenosine deaminase (ADA), interferon gamma (IFN-*γ*), and a variety of tumor markers and cytokines have been proposed as alternative noninvasive means of establishing tuberculous etiology [4]. ADA is an enzyme involved in purine catabolism, catalyzing the pathway from adenosine to inosine and is known as a cellular immunity marker. ADA activity has been assessed in various fluids of TB patients for diagnosis of pleural, cerebrospinal, peritoneal, and synovial TB [3, 5–7]. To our knowledge, a few studies [8–11] have evaluated BALF ADA activity for the diagnosis of TB and the results are variable. Therefore, the aim of this study was to calculate the cut-off point for ADA activity in the BALF of patients with TB in a local Iranian population.

The article "Predictive Role of ADA in Bronchoalveolar Lavage Fluid in Making the Diagnosis of Pulmonary Tuberculosis" was retracted in 2014. Reasons: plagiarism; overlap with other authors' work.

## 2. Materials and Methods

A cross-sectional descriptive study was performed at the Shahid Sadoughi Hospital in Yazd, Iran, between 2009 and 2010. This work has been carried out in accordance with the Declaration of Helsinki (2000) of the World Medical Association. This study was approved by the university ethics committee, and then the forms for recording demographic data were completed.

To detect differences in BAL ADA levels between patients with TB and those in control group as has been shown previously in Kayacan et al. [8] study, with a two-sided 5% significance level and power of 80%, a sample size of at least 14 patients in each group was needed.

Sixty-three patients suspected of having pulmonary TB with negative sputum smears for AFB or who had other indications for bronchoscopy were included in the study. Exclusion criteria were as follows: (1) arterial hypoxia, (2) uncooperative patients for bronchoscopy, (3) refractory hypoxia, (4) hemodynamic disorder, (5) life-threatening cardiac arrhythmia, (6) known TB cases (possessing positive sputum test). Sputum samples of all patients were sent to the laboratory for TB culture. A written consent was obtained from each patient and after 4 h fasting and local administration of lidocaine 2% spray, a fiberoptic bronchoscopy (Olympus bronchoscope type 1T20, Japan) was done. BAL fluid was obtained from a pulmonary lobe with the most involvement seen on chest X-ray and a right middle pulmonary lobe in patients with a diffuse involvement or a normal chest X-ray. To obtain BAL fluid, 150 cc normal saline was injected and the returned fluid was collected via a suction and sent to the laboratory for AFB smear and culture. To assess ADA activity, the samples were centrifuged and kept at −21°C. Then ADA levels in BAL fluids were compared to each other by ADA kit (Shim Enzyme CO.). ADA activity was measured by Giusti's colorimetric method. In Giusti's the first step is deamination of adenosine and releasing ammonia. The second reaction is catalyzed by glutamate dehydrogenase accompanying an allosteric activator. Low light absorption at 340 nm has a direct relationship to ADA activity. By this method, ADA activity can be measured up to 100 IU/L. Those patients who had positive sputum cultures or BAL cultures for AFB were selected as the pulmonary TB group; those who had other forms of pulmonary diseases and were negative for TB were included in the non-TB lung disease group. Individuals, in which TB and other pulmonary diseases were ruled out, were selected as the control group. Questionnaires were filled for all three groups and mean ADA levels in BAL fluids were measured and compared. Data were analyzed by independent *t*-test, ANOVA, and Fisher's exact test using SPSS software ver. 11.5.

The article "Predictive Role of ADA in Bronchoalveolar Lavage Fluid in Making the Diagnosis of Pulmonary Tuberculosis" was retracted in 2014. Reasons: plagiarism; overlap with other authors' work.

## 3. Results

Sixty-three patients were enrolled in this study. Fifteen patients (5 males, 10 females; mean age: 64.06 ± 19.37 years) had pulmonary TB, 33 (22 males, 11 females; mean age: 56.18 ±18.60 years) had non-TB lung disease, and 15 cases (10 males, 5 females; mean age: 42.13 ± 21.45 years) were controls. Among non-TB lung disease patients, 5 patients had interstitial lung disease (1 Wegener's disease, 2 cases of usual interstitial pneumonia, 1 case of sarcoidosis, and 1 silicosis), 14 had lung cancer (6 adenocarcinomas, 4 squamous cell carcinomas, 1 small cell carcinoma, 2 non-Hodgkin's lymphomas, and 1 primary pulmonary Hodgkin's lymphoma), 4 had pneumonia, and 10 patients had chronic obstructive pulmonary disease (COPD). Control subjects undergoing bronchoscopy for various reasons and no pathologic findings could be reached eventually. Sputum culture, BAL smear, and BAL culture were positive in 5, 8, and 11 patients, respectively, in pulmonary TB group. As a whole, all TB patients had positive sputum culture or positive-BAL culture (Table 1). In the two other groups, sputum smear and culture and BAL culture were negative for TB. ADA levels in BAL fluids of pulmonary TB group, non-TB lung disease group, and control group were 4.13 ± 2.55 IU/L, 2.42 ± 1.06 IU/L, and 1.93 ± 0.88 IU/L, respectively. One-way ANOVA showed a significant difference in mean ADA level among the 3 groups (*P* = 0.000).

Tukey's test also showed a significant difference between TB patients and non-TB lung disease group (*P* = 0.02) and also TB patients and the control group (*P* = 0.01), but no significant difference was detected between non-TB lung disease patients and the control group (*P* = 0.55) (Table 2). Based on the results, ADA level was 2.43 ± 1.23 IU/L in women and 3.11 ± 2.17 IU/L in men; independent *t*-test did not show a significant difference between the two groups (*P* = 0.11, *t* = 1.58). To determine the best predictive value of ADA levels in diagnosis of pulmonary TB, a ROC curve was used which did not show a significant difference (*P* = 0.10). At the designated cut-off level of 3.5 IU/L, the highest sensitivity and specificity for diagnosis of TB were found (specificity = 84%, sensitivity = 57%). Using cut-off point in ADA = 2.2 IU/L (mean ADA + 2 × SD) in the control group, the sensitivity, specificity, positive-predictive, and negative-predictive values were 73%, 67%, 41%, and 89%, respectively.

The article "Predictive Role of ADA in Bronchoalveolar Lavage Fluid in Making the Diagnosis of Pulmonary Tuberculosis" was retracted in 2014. Reasons: plagiarism; overlap with other authors' work.

## 4. Discussion

Our findings showed a significant difference in ADA levels among three groups and ADA level was significantly higher in TB patients than in the other two groups. ADA is an enzyme that increases in TB because of the stimulation of T-cell lymphocytes by mycobacterial antigens. Since 1978, when ADA activity was found to be high in tuberculous exudates [12], ADA has been used in the diagnosis of tuberculosis [13, 14]. The laboratory method for measuring ADA is inexpensive and relatively simple to perform. Thus, it may be useful in laboratories with limited resources, particularly in developing countries such as Iran. Orphanidou et al. [11] compared ADA activity and lysozyme levels in BAL fluid of smear-negative pulmonary TB patients and non-TB lung disease patients and found that there was no significant difference in lysozyme level of BAL fluids between the two groups, but ADA level in BAL fluids of pulmonary TB patients was significantly higher than that of non-TB lung disease patients (*P* < 0.001). In a study conducted by Kubota et al. [10] mean ADA level in BAL fluid of miliary TB patients, sarcoidosis patients, idiopathic interstitial pneumonia patients, and control group was 5.02 ± 3.75 IU/L, 1.06 ± 0.99 IU/L, 0.21 ± 0.43 IU/L, and 0.3 ± 0.51 IU/L, respectively, and ADA level in BAL fluid of miliary TB patients was higher than that of other groups (*P* < 0.01). In a study by Kayacan et al. [8], ADA level in BAL fluids of pulmonary TB patients, non-TB lung disease patients (like interstitial lung disease, lung cancer, pneumonia, and COPD) and controls was 3.1 ± 2 IU/L, 0.4 ± 0.5 IU/L, and 0.2 ± 0.4 IU/L, respectively, (*P* < 0.001). However, Reechaipichitkul et al. [9] compared ADA levels in BAL fluid of pulmonary TB patients, lung cancer patients, and those with other forms of pulmonary diseases and found no significant difference among these three groups (*P* = 0.56).

Orphanidou et al. [15] showed that ADA level in BAL fluid of patients with pulmonary TB is significantly higher than that of other pulmonary diseases. On the other hand, Boonsarngsuk et al. [16] revealed that BALF ADA had limited value in differentiating pulmonary TB from some other pulmonary diseases. To explain these discrepancies, differences between reported ADA levels and their sensitivity and specificity in different studies, it must be considered that it may be due to different methods of ADA measurement, presence of other diseases, and differences in the technique of bronchoalveolar lavage. In addition, BAL fluid ADA activity may differ from one human race to another [17]. It seems, therefore, that the cut-off value should be ideally based on the results of local studies or studies performed in similar populations and with the same methodology. TB epidemiology is also important. It should be noted that the value of any diagnostic test has been related to its disease prediction ability. Positive predictive value (PPV) in diagnostic studies is related to disease prevalence and thus in population with lower prevalence we suspected to have low PPV. On the other hand it should be remembered that the predictive value of ADA depends not only on its sensitivity and specificity but also on the local prevalence of the disease. When the prevalence rose, the PPV increased [18]. The opposite relation refers to negative predictive value (NPV). Furthermore, most studies are on the total ADA level, but ADA isoenzymes may be more accurate. We were unable to determine ADA isoenzymes. However, in this study at the designated cut-off level = 3.5 IU/L, a specificity = 84% was obtained which indicated that ADA > 3.5 IU/L can confidently rule out non-TB pulmonary diseases.

The article "Predictive Role of ADA in Bronchoalveolar Lavage Fluid in Making the Diagnosis of Pulmonary Tuberculosis" was retracted in 2014. Reasons: plagiarism; overlap with other authors' work.

In conclusion, although ADA level in BAL fluid of patients with pulmonary TB is significantly higher than that of other pulmonary diseases and is a rapid and cost-effective method, its sensitivity is not able to rule out pulmonary TB. Therefore, studies with a larger sample size are recommended.

## Figures and Tables

**Table 1:** Frequency of patients with pulmonary TB based on sputum smear sputum culture and BAL culture.

	Smear		Culture	
	Negative	Positive	Negative	Positive
Sputum *N* (%)	15 (100%)	0 (0%)	10 (67%)	5 (33%)
BAL fluid *N* (%)	7 (47%)	8 (53%)	4 (27%)	11 (73%)

**Table 2:** Mean and SD of ADA level in BAL of patients in 3 study groups.

	Mean ± SD	Maximum	Minimum
Pulmonary TB	4.13 ± 2.55	10	1
Non-TB lung disease	2.42 ± 1.06	5	1
Control	1.93 ± 0.88	4	1
